# Enhanced Translation of mRNAs Encoding Proteins Involved in mRNA Translation during Recovery from Heat Shock

This article has been retracted.

**DOI:** 10.1371/journal.pone.0064171

**Published:** 2013-05-16

**Authors:** Andrea-Kaye Datu, Jnanankur Bag

**Affiliations:** University of Guelph, Department of Molecular & Cellular Biology, Guelph, Ontario, Canada; Tel Aviv University, Israel

## Abstract

The mRNAs encoding poly (A) binding protein (PABP1), eukaryotic elongation factor 1A (eEF1A) and ribosomal protein S6 (RPS6) belong to the family of terminal oligo pyrimidine tract (TOP) containing mRNAs. Translation of the TOP mRNAs is regulated by growth signals and usually codes for proteins involved in mRNA translation. Previous studies from our laboratory showed that translation of PABP1 mRNA was preferentially enhanced during recovery of HeLa cells from heat shock. Presence of the 5′ TOP *cis* element was required for the observed increase of PABP1 mRNA translation. In the studies reported here we showed that translation of two additional TOP mRNAs such as, eEF1A and RPS6 was similarly enhanced during recovery. In addition, we showed by *in vivo* cross-linking experiments that the cellular nucleic acid binding protein ZNF9 binds to all three TOP mRNAs examined in these studies as well as to the β-actin mRNA that lacks a TOP *cis* element. Binding of ZNF9 to mRNAs was observed in both heat-shocked and non heat- shocked cells. However, depletion of ZNF9 by siRNA prevented the preferred stimulation of PABP1, eEF1A and RPS6 expression during recovery from heat shock. There was no detectable effect of ZNF9 depletion on the basal level of expression of either β-actin or PABP1, eEF1A and RPS6 in HeLa cells following recovery from heat shock.

**Conclusion:**

Although the presence of ZNF9 was required for the translational stimulation of PABP1, eEF1A and RPS6 mRNAs, the mechanistic details of this process are still unclear. Since ZNF9 was shown to bind both TOP and non-TOP mRNAs, it is uncertain whether ZNF9 exerts its stimulatory effect on TOP mRNA translation following recovery from heat shock through the TOP *cis*-element. Perhaps additional factors or post-translational modification(s) of ZNF9 following heat shock are necessary for the preferred increase of TOP mRNA translation.

## Introduction

PABP is a multifunctional and ubiquitous mRNA-binding protein in eukaryotes.

PABP is known to play a role in several cellular processes including stimulation of mRNA translation and control of mRNA stability [1] [2]. As such, PABP is important for cell survival. PABP has also been seen to play a role in development and in cancer [3] [4] [5]. Almost all known functions of PABP are attributed to its ability to bind to the poly (A) tail and to act as a scaffold for protein-protein interactions [6]. The other members of cytoplasmic PABP family are t-PABP also known as PABP2 in mouse and PABP3 in humans, PABP4 (or inducible PABP) and PABP5 are separate gene products but are highly homologous to PABP1. All four cytoplasmic PABPs have four RNA binding domains at their N-terminal ends and with the exception of PABP5, have a proline rich linker and a PABPC domain [7]. PABP5 is a smaller polypeptide than all other cytoplasmic PABPs and is missing the entire C-terminal end. Very little information regarding the biochemical functions of these cytoplasmic PABPs are known. Antisense morpholino oligodeoxynucleotide mediated knock down experiments in *Xenopus laevis* suggests that both PABP1 and PABP4 are required for normal development [8] [9]. In addition, rescue studies [8] showed that PABP4 could not restore the effect of PABP1 knock down on development. Therefore, it is likely that each PABP has distinct functions in vertebrates [8]. PABP1 mRNA is a member of the family of mRNAs containing a terminal oligo pyrimidine tract (TOP) at their 5′ ends [10]. TOP mRNAs are growth-dependent mRNAs and encodes various components of the translation apparatus such as several ribosomal proteins and the elongation factors eEF1A and eEF2 [11]. The TOP *cis*-regulatory element typically starts with a C residue at the cap site followed by a stretch of 4–14 pyrimidines and is generally composed of a similar proportion of C and U residues which is trailed by a CG rich sequence. In mammals, the activity of TOP is contained within the first 30 nucleotides of TOP mRNAs and is strictly dependent on its integrity adjacent to the cap structure; therefore it fails to have any effect on mRNA translation when it is located internally even when it comes before an A residue [12].

The translation of TOP mRNAs is sensitive to the cellular growth rate. Thus, arrest in cell growth results in inhibition of TOP mRNA translation. This is observed by their shift from polysomes in growing cells into free mRNP particles (sub-ribosomal fraction) in quiescent cells [12]. These TOP mRNAs are maintained in a repressed state for later use when better growth conditions return. This bimodal distribution of TOP mRNAs between mRNP and polysomes suggests that the translational repression results from an obstruction at the translational initiation step [11].

Translational control of TOP mRNAs allows cells to quickly repress the biosynthesis of translational machinery during episodes of amino acid shortage resulting in growth arrest and thus preventing unnecessary energy wastage [12] [13]. The detailed mechanism of translational control of different TOP mRNAs may be different. It has been observed that there may be a relationship between the phosphorylation of ribosomal protein S6 (RPS6) by p70 ribosomal protein S6 kinase 1 and translational activation of TOP mRNAs [11]. RpS6 is phosphorylated by S6K (S6 kinase) 1 and 2 in response to mitogens. When S6K activity is blocked using the mTOR (mammalian target of rapamycin) inhibitor, rapamycin, there is repressed translation of TOP mRNAs in N1H 3T3 cell lines [14].

However this model remains controversial. A study using amino acid starved cells, which results in the translational repression of TOP mRNAs, observed that RPS6 phosphorylation is insufficient to relieve the translational repression of TOP mRNAs [15]. Another study using mice showed that translation of TOP mRNAs still occurs when mice lack both S6K genes [16]. It is however possible that different strategies are employed by cells to stimulate TOP mRNA translation under different circumstances.

It has been suggested that the 5′ TOP motif is recognized by specific *trans*-acting factors that have the ability modulate TOP mRNA translation. An example of a *trans*-acting factor is the La auto antigen protein which is an RNA-binding protein that is involved in initiation and termination of RNA polymerase III transcription. A study using *Xenopus* cell lines with inducible over-expression of wild-type La or a mutated La, suggested that the La protein also plays a positive role in translation of TOP mRNAs. It was shown that it had a stimulatory effect on the translation of TOP mRNAs including those encoding several ribosomal proteins and eEF1A [17]. Furthermore, another study investigated the translational control of TOP mRNA encoding eEF1A in rapamycin treated human BJAB B lymphocytes. Gel shift assays confirmed that La interacts with an RNA containing the eEF1A TOP element. However, using a functional *in vitro* assay, it was observed that recombinant La protein specifically repressed expression of a reporter mRNA that contained the EF1A TOP element [18]. Collectively, these results indicate that TOP mRNA translation may be either repressed or activated through La binding to the TOP element.

More recently, the presence of another TOP binding protein has been reported. Myotonic dystrophy 2 (DM2) is a disease of the skeletal muscle and is caused by (CCTG)n expansion in the introns 1 of the *ZNF9* (Zinc finger factor 9) gene, also known as the cellular nucleic acid binding protein (CNBP). The ZNF9 protein contains 7 zinc finger domains and is believed to function as an RNA-binding protein [10]. Its absence in DM2 cells is thought to contribute to the disruption of RNA metabolism in these cells [19]. The biological function of ZNF9 in normal and DM2 cells is not entirely clear. ZNF9 structure is highly conserved suggesting that this protein plays a basic biological role [10]. The seven conserved Zinc-finger (CCHC) repeats are found commonly in transcription factors, ribosomal proteins, and proteins involved in the processing of mRNAs coding for ribosomal proteins [10]. Several studies suggested a role of ZNF9 in regulating both cap-dependent and cap-independent translation [19] [20]. ZNF9 has been shown to bind the internal ribosome entry site (IRES) *cis* element of human ornithine decarboxylase (ODC) mRNA and forms an IRES trans-acting factor complex with another known IRES binding protein PCBP2. Mutational studies of IRES of ODC mRNA showed that mutations that abolished IRES function also reduced binding to ZNF9 and PCBP2 [20]. Both human and Xenopus laevis ZNF9 can bind to TOP elements of several mRNAs including eEF1A, eEF2, RPS17, RPL4 and PABP1 [10] [19]. Binding of ZNF9 to these mRNAs is believed to stimulate their translation. It was reported that there is reduced expression of ZNF9 in myotonic dystrophy patients which leads to a decrease in translation of TOP mRNAs as well as of global mRNA translation [10]. It is not clear whether the decline of global mRNA translation was due to the effect of ZNF9 depletion on the reduced translation of several TOP mRNAs encoding various factors necessary for mRNA translation. Furthermore, as expected ectopic expression of ZNF9 in DM2 myoblasts resulted in an increased rate of protein synthesis, suggesting that stimulation of translation of TOP mRNAs was responsible for the observed effect on global protein synthesis in DM2 muscle cells [10]. The details, however, of how ZNF9 or any other novel TOP binding protein enhances translation remains to be investigated.

In our laboratory we have used heat shock treatment to study regulation of TOP mRNA translation [21]. It is well known that translation of normal cellular mRNAs undergoes rapid changes when cells are subjected to heat shock. Cells down regulate protein synthesis in order to cope with stress [22], because the presence of many unfolded proteins produced by heat shock may harm the survival of cells which could ultimately lead to cell death.

The precise mechanism of how general cap dependant cellular mRNA translation is inhibited in heat-shocked cells is not fully understood. Most likely, it takes place through inactivation of the eIF4F complex and other initiation factors. Studies have shown that there is decreased phosphorylation of eIF4E and eIF4B, increased phosphorylation of eIF2α, and insolubilization of eIF4G following heat shock [21]. Since PABP1 interacts with eIF4G, regulation of its expression is important in modifying gene expression in response to heat stress. Studies from our laboratory have shown that indeed there was a decline in the cellular abundance of PABP1 following 2 hours of heat shock in HeLa cells. However, during the recovery period in which the cells were placed back to their normal temperature following heat shock, PABP1 abundance increased 2.5 fold [21]. This increase in PABP1 abundance during recovery from heat shock was achieved by translating PABP1 mRNA more efficiently. It was postulated that the increase in PABP1 abundance may act as a signal for cells to stimulate global mRNA translation to meet protein synthesis requirements for the cell to recover completely from the heat induced stress. Results from our laboratory showed that the TOP *cis*-element of PABP1 mRNA is responsible for the preferential increase of PABP1 mRNA translation in cells undergoing recovery from heat shock [21].

In this report we examined whether translation of other TOP mRNAs such as RPS6 and eEF1A are also up regulated during recovery from heat shock and investigated the nature of the trans-acting factor responsible for regulating translation of TOP mRNAs in HeLa cells. We demonstrate here that expression PABP1, eEF1A and RPS6 mRNAs were enhanced during recovery from heat shock. We showed that ZNF9 interacts with both TOP^+^ and non TOP^−^ cellular mRNAs. However, depletion of ZNF9 abolished the preferred increase of PABP1, eEF1A and RPS6 expression during recovery from heat shock. Our results suggest an essential role of ZNF9 in the stimulation of translation during recovery from heat shock of all three TOP mRNAs examined here.

## Materials and Methods

### Cell Culture and Heat Shock Treatment

HeLa cells were grown at 37°C with 5% CO_2_ in Dulbecco’s Modified Eagle Medium (DMEM) supplemented with 10% fetal bovine serum (FBS) for 2–3 days to desired confluence. Cells were subjected to heat shock at the indicated temperatures for different times, and returned to 37°C for recovery. Control cells were maintained at 37°C.

### Western Blotting

Cells were washed three times with 1×PBS (125 mM NaCl, 1.5 mM KH_2_PO4, 8 mM Na_2_HPO4 and 2.5 mM KCl) and lysed with 200 µL of 1× SDS gel-loading buffer (50 mM Tris-HCl, pH 6.8; 2% (w/v) SDS; 0.1% (w/v) bromophenol blue; 10% (v/v) glycerol and 5% (v/v) 2-mercaptoethanol). The samples were boiled for 5 minutes and 10 µL aliquots were separated by 10% SDS-PAGE. The separated polypeptides were electrophoretically transferred from the gel onto a nitrocellulose membrane. Afterwards, membranes were blocked with a blocking buffer (5% non fat dry milk, 0.2% Tween-20 in PBS) for 3 hours at room temperature. Proteins were detected by incubating the membrane with the appropriate specific primary antibody (Table 1) for 2–4 hours at room temperature, followed by incubation with the appropriate HRP-conjugated secondary antibody. The membrane bound antigen-antibody complex was developed with western lighting chemiluminescence reagent plus (PerKinElmer, LAS, Inc. Shelton, USA). The X ray film was scanned and quantified by using the Image J program and recorded in arbitrary units after subtracting the background.

**Table 1:** Primary antibodies used for immuno blotting.

Type	Name	From (Company)
Primary	β – actin	Santa Cruz Biochemical, Santa Cruz, CA, USA
Primary	PABP	Santa Cruz Biochemical, Santa Cruz, CA, USA
Primary	PABP 3	Abnova, Wal Nut, CA, USA
Primary	PABP 4	Novus Biologicals, ON, Canada
Primary	PABP 5	Santa Cruz Biochemical, Santa Cruz, CA, USA
Primary	HSP 70	Santa Cruz Biochemical, Santa Cruz, CA, USA
Primary	eIF2α	Santa Cruz Biochemical, Santa Cruz, CA, USA
Primary	Paip1	Abcam, SF, CA, USA
Primary	eEF1A	Cell Signaling Tech., Danvers, MA, USA
Primary	RPS6	Abnova, Wal Nut, CA, USA
Primary	ZNF9	Abcam, SF, CA, USA
Secondary	Anti-mouse	Santa Cruz Biochemical, Santa Cruz, CA, USA
Secondary	Anti-rabbit	Santa Cruz Biochemical, Santa Cruz, CA, USA
Secondary	Anti-goat	Santa Cruz Biochemical, Santa Cruz, CA, USA

### RT PCR

Cells were washed three times with 1×PBS and total cellular RNA was isolated using the High Pure RNA Isolation Kit according to manufacture’s instructions (Roche Biochemical, Indianapolis, IN, USA). The quality and quantity of the RNA were determined by 1.5% agarose gel electrophoresis and spectrophotometric measurements respectively. The absence of contaminating DNA in RNA samples was tested by PCR using several mRNA specific primers. The levels of specific mRNAs were determined by RT-PCR. An aliquot of total RNA (500 ng) was reverse transcribed at 42°C for 1 hour in a total reaction volume of 20 µL using SuperScript II reverse transcriptase (Invitrogen, Burlington, Canada) and 150 ng of random primers. After the reaction, 2 µL of the cDNA sample was amplified by PCR in a total master mix (Fermentas, Amherst, NY, USA) reaction volume of 50 µL, which included 100 ng of primers specific for PABP1, β –actin, eEF1A1, eEF1A2 or RPS6 (Sigma, Oakville, ON, Canada) (Table 2). The amplification was performed using an initial denaturation step at 95°C for 4 min, and for the mRNAs measured in this study, was followed by 25 cycles of denaturation at 95°C for 20 s, annealing ranging from 58–66°C, depending on the primer for 20 s and extension at 72°C for 20 s. Samples from the PCR reactions were analyzed by 1% agarose gel electrophoresis and the band intensities of the scanned images of the print were quantified by using the Image J program. The relative expression values of all mRNAs were normalized to the β-actin mRNA level. For detecting any DNA contamination of our RNA, PCR reactions of each RNA samples were carried out without the reverse transcription step.

**Table 2:** Primers used for RT-PCR. S, sense oligonucleotide; AS, antisense oligonucleotide.

mRNA	Nucleotide Sequence (5′ to 3′)
Human β –actin (S)	CTCTTCCAGCCTTCCTTCCT
Human β –actin (AS)	CACCTTCACCGTTCCAGTTT
PABP1 (S)	GCACAGAAAGCTGTGGATG
PABP1 (AS)	TTTGCGCTTAAGTTCCGTC
eEF1A1 (S)	GGCATACCCGAGAGCATG
eEF1A1 (AS)	AGGCAT GTTAGCACTTGGC
eEFA2 (S)	GAGCCCTCCCCCAACATGCC
eEFA2 (AS)	ATGTTCACTGGCGCAAAGGTCAC
RPS6 (S)	GTTATCTGCTGACTGCCTTGGA
RPS6 (AS)	GGGAATCCCTGTTTGTCGTTT

### Immunoprecipitation of RNA-Protein Complexes

RNA-protein cross-linking and immunoprecipitation assay was performed as previously described in [23]. Cells in a 35 mm dish were treated with 1% formaldehyde (Electron Microscopy Sciences) in PBS for 30 minutes at room temperature to crosslink the RNA and proteins of RNP complexes. Cells were then incubated in 0.25 M of glycine for 15 minutes which was removed before cell lysis. Cells were then removed from the plate using a scraper with 0.1 mL of RIPA buffer (50 mM Tris-HCl, 1% Ipegal CA6–30, 0.5% sodium deoxycholate, 0.05% SDS, 1 mM EDTA, 150 mM NaCl, 0.5 mM PMSF, 10 µg/mL leupeptin, 2 µg/mL aprotinin, 100 U RNasin (Promega). The cell suspension was passed through a 20 gauge syringe several times until more than 90% of cells were lysed as judged by phase contrast microscopy. The cell lysate was centrifuged at 10, 000 rpm for 1 minute in a microfuge at 4^°^ C. The supernatant was first pre-cleared by mixing with a 20 µL packed volume of Sepharose G and 100 µg of *E.coli* t-RNA in a rotator for 1 h at 4°C. It was then centrifuged at 4000 rpm for 5 minutes and the supernatant (cell lysate) was collected. ZNF9 (Abcam, San Francisco, CA, USA) antibody and 10 µg coated protein G-Sepharose beands (20 uL, packed volume) was incubated with the pre-cleared cell lysate (100 uL) in RIPA buffer at 4°C for 2 hours. The beads were washed extensively with high-stringency RIPA buffer (50 mM Tris-HCl, 1% Ipegal CA-630, 0.1% sodium deoxycholate, 0.1% SDS, 1 mM EDTA, 1 M NaCl, 2.5 M Urea and 0.5 mM PMSF) five times for 10 minutes at room temperature. The RNA-protein cross-links were reversed by incubation at 70°C for 45 minutes in 100 µL of elution buffer (50 mM Tris-HCl, 5 mM EDTA, 10 mM DTT, 1% SDS). The RNA was then extracted with three volumes of a mixture of phenol/chloroform (50/50). The RNA was precipitated using one volume of ethanol, and left overnight at −20°C. The precipitated RNA s was collected by centrifugation at 6000 rpm for 10 minutes at 4°C and resuspended in RNAse free water. Contaminating DNA was removed from the samples by RQ1 RNase-free DNAse (Promega) treatment prior to being reverse transcribed using random primers as described above followed by PCR amplification using specific primers (Table 2). The samples were analyzed by electrophoresis in a 1% agarose gel and band intensities were determined by scanning and Image J program analysis and expressed as arbitrary unit after normalizing by the β-actin mRNA level.

### Sub-cellular Fractionation of Polysomes and RNA Isolation

Samples corresponding to equal numbers of cells were used for analysis. The cells were lysed in 500 µL of polysomal buffer (10 mM MOPS, pH 7.2, 250 mM NaCl, 2.5 mM MgOAc, 0.5% Nonidet P-40, 0.1 mm phenylmethanesulfonyl fluoride, 200 µg mL^−1^ heparin, and 50 µg mL^−1^ cycloheximide) [24]. After removal of the nuclei and cell debris by centrifugation at 12,000 x g for 10 min, the supernatant fraction was centrifuged in a 12 mL 10–50% sucrose gradient, containing 25 mM Hepes (pH 7.0), 50 mm KCl, 2 mM MgOAc, 200 µg mL^−1^ heparin, 50 µg mL^−1^ cycloheximide and 15 mM 2-mercaptoethanol at 100,000 x g in a Beckman SW 41 Ti rotor for 3 h. Gradient fractions of approximately 1 mL each were collected using an Auto Densi-Flow IIC apparatus (Buchler Instruments, Fort Lee, NJ, USA) [24]. Fractions 1–3, 4–6 and 7–10 were pooled together and total RNA from each fraction was isolated using Trizol as described by the manufacturer (Roche), and precipitated with ethanol. Absence of contaminating DNA in RNA samples was examined by PCR using several mRNA specific primers.

### Cell Culture and siRNA Transfection

HeLa cells were grown at 37°C in Dulbecco’s modified Eagle’s medium (DMEM) supplemented by 10% fetal bovine serum (FBS) for 2–3 days, until the desired degree of cell confluence was obtained. One day before transfection, cells were trypsinized and suspended in 1 mL of DMEM medium. 100 µL of suspended cells were grown in a 35 mm tissue culture dish with 2 mL of DMEM medium including 1% glutamine (Sigma, Oakville, Canada) and 10% fetal bovine serum (VWR, Mississauga, ON, Canada) without antibiotics in a humidified 5% CO_2_ incubator at 37°C. Cells were either kept at 37°C as controls or were heat shocked for 3 hours at 44°C and allowed to recover for 4 hours at 37°C. Control and recovered cells were transfected at 30–50% confluence using Lipofectamine 2000™ (Invitrogen, Burlington, ON, Canada). For each transfection, 1.5 µL of siRNA duplex (20 µM annealed duplex from Invitrogen) was mixed with 250 µl of OPTI-MEM® I (Invitrogen, Burlington, ON, Canada). In a separate tube, 5 µL of Lipofectamine 2000™ was diluted with 250 µL OPTI-MEM® I and incubated for 5 minutes at room temperature. Afterwards, both solutions were mixed gently and incubated for 20 minutes at room temperature to form a complex. The solutions were then added to the 35 mm dish containing cells and 1 mL of medium. Cells were incubated at 37°C in a CO_2_ incubator in presence of the transfection complex for 24 hours, then the media was refreshed and kept at 37°C for 20 hours and then processed for further analyses. All cell samples were transfected with either anti CNBP siRNA (siZNF9) or a validated negative control siRNA from Qiagen (Cambridge, MA, USA). Additionally non-transfected cells and mock transfected cells were used as controls. The sequence of the ZNF9 siRNA and control siRNA are:

3′-ACAGCGAUAACAAAUAUCUgg-5′ and 5′-AGAUAUUUGUUAUCGCUGUtt -3′; 5′-UUCUUCGAACGUGUCACGUdTdT and 5′-ACGUGACACGUUCGGAGAAdTdT-3′. For mock transfection, cells were treated with the transfection reagent without the siRNA for the same length of time as transfection with siRNA.

## Results

### Expression of Polypeptides Involved in Translation During Heat Shock and Recovery

Previously we reported that translation of PABP1 mRNA is preferentially enhanced in HeLa cells during recovery from heat shock at 37°C [21]. PABP1 mRNA belongs to a family of TOP containing mRNAs that include mRNAs encoding various components of the cellular translation machinery such as eEF1A, and different ribosomal proteins. We therefore examined whether eEF1A and ribosomal protein S6 (RPS6) are co-coordinately regulated with PABP1 during recovery from heat shock. The abundance of three polypeptides, PABP1, eEF1A (both A1 and A2 isoforms) and RPS6 following heat shock and recovery was measured by western blotting (Figure 1A). Prior to these analyses the conditions of western blotting was optimized for linear dose response (Figure 1B). These polypeptides showed a differential effect of heat shock on their abundance. Abundance of PABP1 was significantly reduced by heat shock while that of eEF1A and RPS6 remained virtually unchanged. However, following recovery, levels of all of these polypeptides increased by almost 2 fold over what was observed in the non-heat shocked control cells. We also tested whether the abundance of another translation initiation factor such as eIF-2α and a translation regulatory protein Paip1 responds similarly to heat shock. The abundance of eIF-2α did not change after heat shock but that of Paip1 showed a decrease similar to what was observed for PABP1 (Figure 1A). Since Paip1 is a PABP1 interacting protein, it is not surprising that the cellular levels of both proteins are coordinately regulated. However, in contrast to PABP1, eEF1A and RPS6, the abundance of Paip1 and eIF-2α did not increase following recovery. In our studies cellular β –actin level was used as a control and its cellular level did not change significantly following heat shock and recovery.

**Figure 1:** Changes in cellular level of polypeptides during heat shock and recovery. A) Cells were grown to 40% confluence and heat shocked for 3 hours at 44°C and recovered at 37°C for 24 hours. The control cells were maintained at 37°C. For all experiments cells were directly lysed on the plate using gel loading buffer, and lysates were analyzed by SDS/PAGE. Individual polypeptides were detected by western blotting using appropriate antibodies. B) Shows dose response of western blotting of cell extract from exponentially growing cells with different antibodies. The sample volumes are indicated at the top of the panel. The abundance of specific polypeptides in both panels was determined by scanning the X-ray film and quantifying the images with Image J as described in materials and methods. The values in arbitrary scale are shown bellow each lane. All values were normalized by the using the β -actin levels as loading controls. The experiment was repeated three times, and the averages are shown in panel B as mean ± standard error. C) Western blotting and quantification was performed to measure the abundance of PABP4 in control, heat- shocked and recovered cells as described above. Data are mean ± SE, p<0.05 for those with an * and p>0.05 for those that are unmarked, n = 3.

In addition to PABP1, PABP4 is also expressed in HeLa cells [25]. Since PABP4 mRNA is not a TOP containing mRNA we examined whether the cellular abundance of PABP4 was influenced by heat shock and recovery. The results show (Figure 1A) that the cellular level of PABP4 remained unchanged by heat shock and did not increase following recovery from heat shock treatment.

### Changes in Specific mRNA Levels following Heat Shock and Recovery

In order to assess whether the increase in the cellular levels of PABP1, eEF1A and RPS6 was due to an increase in the cognate mRNA level, different mRNA levels were measured by RT-PCR (Figure 2). To determine the optimum cDNA concentration and cycle time for a linear dose response, samples were subjected to 25 cycles of amplification with different concentrations of cDNA using different mRNA specific primers. The results show (Figure 2A), that 1.5–3 µL of cDNA samples and 25 cycles of PCR under these reaction conditions were within the linear range of dose response for PABP1, eEf1A1 and 2, RPS6 and β–actin mRNA. Furthermore, no product was observed when reverse transcription step was omitted before the PCR (-RT lane). Minus RT reactions were performed with the same RNA samples used in RT-PCR studies, and all mRNAs were measured using the same cDNA preparation, thus confirming that, the PCR products were derived from RNA. For subsequent studies we used 2 µL of cDNA and 25 cycles for PCR. The results show that the PABP1, eEF1A1, eEF1A2, and RPS6 mRNA levels were not altered by exposure to heat shock or following the subsequent recovery phase (Figure 2B & C). These results suggest selective enhancement of translation of PABP1, RPS6, eEF1A1 and eEF1A2 mRNAs during recovery from heat shock. Both eEF1A1 and eEF1A2 are TOP mRNAs encoded by different genes [26] with tissue specific patterns of expression. eEF1A1 is expressed in the brain, placenta, lung, liver, kidney, and pancreas, while eEF1A2 is expressed in brain, heart, and skeletal muscle [27]. However, in HeLa cells expression of both eEF1A1 and eEF1A2 was detected.

**Figure 2:** mRNA levels of PABP1, eEF1A and RPS6. Total cellular RNA from HeLa cells was isolated and the levels of specific mRNAs were determined by RT-PCR. Products of RT-PCR were analyzed by 1% agarose gel electrophoresis and quantified by scanning as described in materials and methods. Where applicable the relative expression values of all mRNAs were normalized by the β-actin mRNA level The values bellow each lane represent the relative abundance of each mRNA using an arbitrary scale where the level in control cells was considered to be 1.00. A) The dose response of the PCR reaction using 25 cycles of amplification for different mRNAs is shown. B) HeLa cells were grown to 40% cell confluence, heat shocked for 3 hours at 44°C and recovered for 24 hours at 37°C. Total cellular RNA from control, heat -hocked and following recovery from heat shock was analyzed**.** The C (-RT) lane indicates samples of amplification of RNA from control HeLa cells without reverse transcription. C) Experiments were repeated three times, and the averages are shown here as mean ± standard error.

### The Polysomal Distribution of Different mRNA following Heat Shock and Recovery

Comparison of mRNA levels for PABP1, eEF1A and RPS6 between control, heat shocked and recovered cells suggest that expression of these proteins is regulated at the level of mRNA translation. Therefore, the polysomal distribution of these mRNAs was studied to examine whether translation of these mRNAs was activated following recovery from heat shock. Translationally active polysomes and non-translated sub-ribosomal populations of mRNAs were separated by means of sucrose gradient centrifugation, as described in the materials and methods section. For our analyses gradient fractions were pooled into three fractions. Fractions 1–3 represent the sub-ribosomal region of the gradient, fractions 4–6 represent the 80S initiation complexes, disomes, trisomes and small polysomes, while fractions 7–10 represent efficiently translated medium to large polysomes [21]. The results from our analyses show that nearly 40–50% of cytoplasmic PABP1, eEF1A and RPS6 mRNAs were present in the non-translated sub -ribosomal fractions of untreated exponentially growing cells. In contrast, only 10–15% of β-actin mRNA was present in this fraction. Following heat shock, the proportion of non translated mRNAs coding for all four polypeptides (PABP1, eEF1A, RPS6, and β-actin) increased to approximately 40–50% of cytoplasmic mRNA. This was most likely due to repression of global mRNA translation by heat shock [22]. However, the effect of reduced mRNA translation in heat-shocked cells did not affect the abundance of different polypeptides to the same extent (compare β-actin and Paip1, Figure 1A). This was probably due to differential stability of the polypeptides. Following recovery from heat shock translation resumed for all four mRNAs, and the majority of non translated sub-ribosomal constituents of PABP1, eEF1A, and RPS6 were transferred to the actively translated fractions (80S to polysomes) and represented almost 90–100% of the cytoplasmic population (Figure 3 panels A and B). Our results show that compared to β-actin mRNA, the PABP1, eEF1A, and RPS6 mRNAs are inefficiently translated in exponentially growing cells. Following recovery from heat shock, there was a preferential increase in the translation efficiency of all three TOP mRNAs.

**Figure 3:** The polysomal distribution of mRNA following heat shock and recovery. Cell lysates were prepared as described in materials and methods and the 12.000×g supernatant fraction of the cell lysate was centrifuged in a 12 mL 10–50% sucrose gradient at 100,000×g in a Beckman SW 41Ti rotor for 3 h. Gradient fractions of approximately 1 mL each were collected and fractions 1–3, 4–6 and 7–10 were pooled together. Total cellular RNA from each pooled fraction was isolated using the Trizol RNA isolation kit as described in materials and methods. A) The abundance of PABP1, eEF1A and RPS6 and β -actin mRNA levels in each fraction was measured by RT-PCR as described in materials and methods section. Each RNA fraction was also subjected to the PCR step without the prior reverse transcription step to determine DNA contamination in our samples, and none was found (results not shown). The amplicons were analyzed by 1% agarose gel electrophoresis, and quantified by scanning the image as described in materials and methods. B) Representative results of two separate experiments. The distribution of mRNA in the sub-polysomal region (fraction numbers 1–3) and the polysomal region (fraction numbers 7–10) of the gradient was determined by quantifying the mRNA level in each fraction using an arbitrary scale. The value of mean ± standard error was derived from two separate experiments.

### Immunoprecipitation of RNA-ZNF9 Complex

ZNF9 is known to bind to the TOP *cis* element of mRNAs in *Xenopus laevis* and regulate both cap-dependent and cap-independent translation [19] [20]. In addition, it was previously reported that ZNF9 deficiency results in reduced translation of several TOP containing mRNAs in muscle cells from a mouse model of myotonic dystrophy [10]. We therefore, examined whether ZNF9 interacts with PABP1, eEF1A and RPS6 RNAs during recovery from heat shock in a human cell culture model using HeLa cells. The RNA and proteins of cellular RNA-protein complexes were covalently cross-linked *in vivo* with formaldehyde. Following cell the RNA protein complexes were immunoprecipitated with an anti ZNF9 and after reversing the cross-link the RNA was extracted and analyzed for the presence of different mRNAs by RT-PCR.

The results (Figure 4A) show that the ZNF9 did interact with PABP1, eEF1A and RPS6 in untreated exponentially growing cells and remained bound to these mRNAs after heat shock and during recovery. The binding of ZNF9 to these mRNAs did not appear to be specific for TOP containing mRNAs as β-actin and GAPDH mRNAs were also present in the immunoprecipitated samples. Furthermore, there were insignificant differences in the levels of different mRNAs immunoprecipitated by ZNF9 antibody from control, heat shocked and recovered samples (Figures 4A & B). These results suggest that ZNF9 may act as a general RNA-binding protein and may not be directly involved in enhancing translation of PABP1, eEF1A and RPS6 mRNAs. Immunoprecipitation and subsequent RT-PCR experiments using non cross-linked samples show that none of the mRNAs examined were immunoprecipitated without cross-linking from exponentially growing cells (Figure 4C, top row). In addition, western blotting of immunoprecipitated samples from cross-linked control, heat-shocked and recovered samples show that ZNF9 was successfully immunoprecipitated (Figure 4C, bottom row).

**Figure 4:** Immunoprecipitation of RNA-ZNF9 Complex. A) HeLa cells were grown to 40% confluence; heat shocked for 3 hours at 44°C, and allowed to recover at 37°C for 24 hours. Cellular RNA and proteins were cross-linked with formaldehyde and lysed as described in materials and methods. Cell lysates were subjected to immunoprecipitation of RNA-ZNF9 complexes as described in the methods section. RNA from the immunoprecipitates was isolated and reverse-transcribed using random primers followed by PCR amplification using mRNA specific primers. PCR products were analyzed by electrophoresis in a 1% agarose gel and quantified by scanning as described in materials and methods. The levels of different mRNAs were normalized to the level of β-actin mRNA and expressed in arbitrary units below each lane. B) Each set of experiments was repeated three times, and the averages are shown here as mean ± standard error. C) First row; as a negative control immunoprecipitation of non cross-linked cell extract of exponentially growing HeLa cells was performed with ZNF9 antibody and RNA was extracted and used for RT-PCR as described in materials and methods. The results of analyses of RT-PCR products by 1% agarose gel electrophoresis with different mRNA specific primers are shown. The bottom row shows the results of western blotting experiment of immunoprecipitated samples prior to RNA isolation from the lysate of cross- linked control (C), heat shocked (HS) and recovered cells (Re). D) Exponentially growing HeLa cells were subjected to cross-linking as described above and the cell lysate was treated with either, non-immunized serum or GAPDH or PABP1 antibody and the RNA was extracted from the immunoprecipitates. The RNA samples were analyzed for the presence of either PABP1 or β-actin mRNA as described before.

Additional control experiments using PABP1, GAPDH antibodies and non-immunized serum for immunoprecipitation showed that β-actin mRNA was immunoprecipitated by PABP1 antibody (Figure 4D). In contrast, GAPDH antibody and non-immunized serum did not pull down β-actin or PABP1 mRNA. Therefore, immunoprecipitation of mRNAs by ZNF9 antibody suggest a specific interaction between these mRNAs and ZNF9.

### Effect of ZNF9 Depletion on TOP mRNA Translation

In order to test whether ZNF9 has any effect on PABP1 expression, we knocked down ZNF9 expression in HeLa cells by using a ZNF9 specific siRNA. We initially tested the efficacy of siRNA on normal (at 37°C) cells using 24 and 48 hours of transfection. The results show that the designed siRNA was able to inhibit ZNF9 expression by approximately 70% (Figure 5A) within 24 hours in exponentially growing control cells. We then used cells that were heat shocked at 44°C for 3 hours for siRNA treatment. In addition we used normal non- transfected and heat-shocked mock-transfected cells as controls. Analyses of polypeptide levels in total cell extracts by western blotting show (Figure 5B & C) that there was approximately 80% reduction in ZNF9 abundance after 24 hours of incubation with the siRNA, in heat shocked cells. There was no reduction of ZNF9 abundance when cells were transfected with the control siRNA or in mock transfected cells. Cellular levels of β-actin were used as loading controls and its abundance was not affected by siRNA treatments. The results (Figure 5B & C) further show that the characteristic induction of PABP1, eEF1A and RPS6 expression during recovery from heat shock was ablated by depletion of ZNF9. The mock and control siRNA transfected cells, however did exhibit normal induction of expression all of these polypeptides during recovery from heat shock. These results, therefore, suggest that the presence of ZNF9 is required for the increased of abundance of PABP1, eEF1A and RPS6 during recovery from heat shock. However, whether this observed effect of ZNF9 depletion was related to the preferred increase of TOP mRNA translation or the presence of the TOP *cis-*element has not been determined yet.

**Figure 5:** ZNF9 knock down with siRNA. A) Exponentially growing HeLa cells were transfected with ZNF9 siRNA as described in materials and methods for 24 and 48 hours. Samples of total cell lysate from non-transfected (C) and transfected cells following 24 and 48 hours of transfection (SiZNF9) were analyzed for the abundance of ZNF9 and β-actin (loading control) by western blotting. B) Cells at 40% confluency were either kept at 37°C as controls or were heat shocked for 3 hours at 44°C and allowed to recover for 4 hours at 37°C before being transfected with either no RNA (M), ZNF9 siRNA or a validated negative control siRNA. Cells were incubated at 37°C in a CO_2_ incubator in the presence of the transfection complex for 24 hours and following lysis samples were processed for further analyses by SDS-PAGE and western blotting as described in materials and methods. C) The abundance of specific polypeptides was determined by scanning the images, and normalizing the values using the β -actin levels as loading controls as described in materials and methods.

## Discussion

### PABP1, eEF1A and RPS6 Abundance following Recovery from Heat Shock

Our studies not only showed preferential increase of PABP1 expression during recovery from heat shock, but the same was seen for the expression levels of eEF1A and RPS6. This is not surprising considering that previous studies found that the abundance of elongation factors and several ribosomal proteins increased when mRNA is reactivated for translation following growth stimulation of serum starved cells [12]. Interestingly, a number of other factors involved in mRNA translation such as eIF2-α and Paip1, which are coded by mRNAs lacking a TOP *cis* element did not show any change in their abundance in our studies. In addition, previous studies from our laboratory reported that the abundance of other initiation factors such as eIF4G and eIF4E also did not change following recovery from heat shock [21]. This is intriguing because PABP, Paip1 and eIF4G are partners of a multi-protein initiation complex; therefore our results suggest that expression of these proteins is not co-coordinately regulated. We also demonstrated that amongst the two different cytoplasmic PABPs, PABP1 and PABP4, expressed in HeLa cells, only PABP1 abundance increased following recovery from heat shock. Again, interestingly the mRNA encoding PABP4 lacks the TOP *cis* element (Figure 6).

**Figure 6:** Nucleotide sequence of the 5′ end of different mRNA. Sequences were obtained from the NCBI database The TOP *cis* elements are highlighted. The 5′ ends of PABP1, eEF1A1, eEF1A2, RPS6 and RPS17 are shown. Note that both RPS17 and eEF1A2 TOP elements contain a terminal G instead of a terminal C present in PABP1, EEF1A1 and RPS6 mRNAs.

### Translational Control of TOP mRNAs

In an attempt to understand how the abundance of PABP1, eEF1A and RPS6 proteins was increased during recovery from heat shock we demonstrated that this increase in protein abundance occurs without a corresponding increase in the level of cognate mRNAs. This observation ruled out the possibilities of either transcriptional control or regulation of mRNA stability as a means of increasing protein abundance. Our analyses of distribution of mRNAs in sucrose gradients clearly showed that PABP1, eEF1A1, eEF1A2 and RPS6 mRNA translation was preferentially enhanced during recovery from heat shock. In an earlier report from our lab it was shown that the translational activation of PABP1 mRNA following recovery from heat shock was indeed mediated by the TOP element [21]. It was shown that the heat shock and recovery response can be transferred to a reporter mRNA by placing the TOP element for PABP1 mRNA at the 5′ end of the reporter mRNA. In this report we showed that RPS6 and eEF1A mRNAs also behave similarly to PABP1 mRNA in response to heat shock. It should be noted that although mRNAs encoding all three proteins examined here behaved similarly to heat stress, the precise nature of the TOP element differs considerably amongst these mRNAs (Figure 6). However, further studies will be necessary to demonstrate that the TOP *cis* element is also involved in the up-regulation of RPS6, eEF1A1 and eEF1A2 mRNA translation during recovery from heat shock.

### Role of ZNF9 in TOP mRNA Translation

How the TOP *cis*-element regulates mRNA translation has remained elusive for more than a decade. Different laboratories have obtained conflicting results regarding the trans- acting factors involved in binding and regulating TOP mRNA translation. Two stress granule associated factors TIA-1 and TIAR have recently been shown to repress TOP mRNA translation by binding to the 5′ end of TOP element upon amino acid starvation [28]. However, repression and subsequent activation of the TOP mRNAs may involve different sets of factors under different conditions. Studies in *Xenopus laevis* suggest that translation of several TOP- containing ribosomal protein mRNAs is regulated by a complex interaction between three different proteins La, ZNF9, and an unidentified protease sensitive factor [17] [19]. It has been proposed that ZNF9 acts as a repressor and following growth stimulation La relieves this repression [17]. In contrast, another recent study reported ZNF9 to be a stimulator of TOP as well as global mRNA translation [10]. We demonstrated here by RNA CHIP analyses that ZNF9 possibly binds globally to most mRNAs since β-actin mRNA which lacked the TOP element was also immunoprecipitated by the ZNF9 antibody. Our results also showed that ZNF9 does not dissociate from the TOP mRNAs studied here following heat shock, and remained bound to TOP and actin mRNAs during recovery. However, since these mRNAs were not immunoprecipitated when the cross-linking step was omitted suggest that binding of ZNF9 might be transient or requires other proteins to form a complex with mRNA. When we tested the effect of ZNF9 knock down on TOP mRNA translation using three different models, a similar effect was observed on the abundance of all three TOP mRNA encoded proteins. We demonstrated that depletion of ZNF9 prevented the accumulation of PABP1, eEF1A and RPS6 during recovery from heat shock. This change was most likely due to the inability of ZNF9 depleted cells to preferentially stimulate TOP mRNA translation following heat shock and recovery. Depletion of ZNF9 however, did not affect the basal level of expression of all four polypeptides including PABP1, eEF1A, RPS6 and β-actin during recovery from heat shock. Our results thus suggest that although the precise nucleotide sequence of the TOP *cis* element of three different mRNAs examined here are different, they are similarly regulated by ZNF9. Our results also suggest that stimulation of TOP mRNA translation by ZNF9 is not directly mediated by its binding to these mRNAs. It appears that a stimulus such as heat shock is necessary to fine tune ZNF9 interaction with TOP mRNAs. The fine-tuning might involve interaction with a TOP binding polypeptide. It is conceivable that a novel protein may bind to TOP elements following heat shock, which in turn interacts with ZNF9 to promote translation of TOP mRNAs. Additionally, post-translational modification(s) of a novel TOP binding protein or ZNF9 itself following heat shock could promote protein-protein interactions and stimulate TOP mRNA translation. It will therefore be important to further investigate whether ZNF9 is post translationally modified and/or interacts with different polypeptide partners following heat shock.

As discussed earlier PABP mRNA translation is positively regulated by TOP and negatively regulated by ARS *cis* elements [2]. Studies from our laboratory have shown that the TOP element from PABP1 mRNA is sufficient for the up-regulated translation of a reporter mRNA during recovery from heat shock. Furthermore, presence of the ARS, where PABP1 itself binds to repress translation [2], down-stream from the TOP of the reporter mRNA, did not influence the up-regulation of translation during recovery. This observation ruled out the possibility that ZNF9 functions by relieving PABP1 mediated repression of translation.

All known TOP containing mRNAs including PABP1, eEF1A and RPS6 are inefficiently translated in exponentially growing cells. Although we know that PABP1 mRNA translation is negatively regulated by a feed back mechanism by binding of PABP1 to the ARS [2], it is not known whether a similar feed back mechanism also regulates RPS6 and eEF1A translation. Interestingly, control of mRNA translation by its own translation product was first described for the bacterial ribosomal protein L10 mRNA more than three decades ago [29], it is therefore, a possibility worth investigating. In addition, different TOP mRNAs may have unique sets of additional control elements that respond to different growth signals. Therefore, a highly complex set of interactions between different *trans*-acting factors and *cis-*elements may determine the fate of TOP mRNA translation. Thus, regulation of the translation of TOP containing mRNAs is more complex than, for example, that of the ferritin mRNA, which lacks the TOP *cis* element. It is known that ferritin mRNA translation is controlled by modulating the interaction between its iron response *cis* element and a single polypeptide by cellular iron level [30]. This is however expected because ferritin mRNA translation needs to respond to one stimulus, namely the intracellular iron level, where as translation of TOP-containing mRNA must respond to many different stimuli.
